The article "Knockdown of ubiquitin-conjugating enzyme E2T (UBE2T) suppresses lung adenocarcinoma progression via targeting fibulin-5 (FBLN5)" was retracted in 2026. Reasons: concerns about the data; concerns about the results or conclusions.

# Knockdown of ubiquitin-conjugating enzyme E2T (UBE2T) suppresses lung adenocarcinoma progression via targeting fibulin-5 (FBLN5)

**DOI:** 10.1080/21655979.2022.2060162

**Published:** 2022-05-11

**Authors:** Yi Li, Xiaojuan Yang, Dan Lu

**Affiliations:** a Department of Respiration Medicine, People’s Hospital of Shanxi Province, Taiyuan City, PR China; b Department of Respiratory Medicine, Shanxi Medical University, Taiyuan City, PR China

**Keywords:** LUAD, UBE2T, proliferation, metastasis, growth

## Abstract

Lung adenocarcinoma (LUAD) is the main histological type of lung cancer, which is the leading cause of cancer-related deaths. Accumulating evidence has displayed that UBE2T is related to tumor progression. However, its role in LUAD has not been fully elucidated. The expression of UBE2T was detected in LUAD tissues by qRT-PCR, western blotting, and immunohistochemistry. UBE2T shRNAs were transfected into LUAD cells to analyze the consequent alteration in function through CCK-8 assay, Edu assay, transwell assay, and TUNEL staining. The potential mechanism of UBE2T was analyzed through GEPIA and verified using ChIP, EMSA, and GST pull-down assays. Furthermore, a xenograft mouse model was used to assess UBE2T function *in vivo*. Results showed that UBE2T level was significantly elevated in LUAD tissues and high UBE2T expression was associated with poor overall survival and disease-free survival. Results from the loss-of-function experiments *in vitro* showed that UBE2T modulated LUAD cell proliferation, migration, invasion, and apoptosis. The mechanism analysis demonstrated that silence of UBE2T increased FBLN5 expression and inhibited the activation of p-ERK, p-GSK3β, and β-catenin. Moreover, following knockdown of UBE2T, the cell proliferation, migration, and invasion were decreased, and sh-FBLN5 partially reverse the decrease. In *in vivo* experiments, it was found that UBE2T knockdown inhibits the tumor growth in LUAD. Immunohistochemically, there was a reduction in Ki67 and an increase in FBLN5 in UBE2T shRNA-treated tumor tissues. In conclusion, UBE2T might be a potential biomarker of LUAD, and targeting the UBE2T/FBLN5 axis might be a novel treatment strategy for LUAD.

## Highlights

- UBE2T high expression was correlated with the poor prognosis in LUAD patients
- Knockdown of UBE2T inhibited LUAD cell proliferation, migration, and invasion
- UBE2T knockdown increased FBLN5 expression and suppressed ERK/GSK3β pathway
- FBLN5 knockdown abrogated the inhibitory effect of sh-UBE2T on LUAD progression
- Knockdown of UBE2T inhibited tumor growth in vivo

## Introduction

Lung cancer is the leading cause of mortality among all malignancies worldwide [1], of which lung adenocarcinoma (LUAD) is the most common subtype, accounting for 40–50% of lung cancer [2,3]. Although achievements have been made in new therapies for LUAD such as chemotherapy, immunotherapy, and molecular targeted therapy, the prognosis of LUAD is still very poor, with a 5-year survival rate of only 15% [4,5]. Therefore, further study of the molecular mechanisms of LUAD is essential for the development of new therapies against LUAD.

Ubiquitin-proteasome pathway (UPP) plays an important role in plant growth regulation, animal reproductive development, tumorigenesis and neurological diseases. E1, E2 and E3 enzymes are involved in ubiquitination progression, of which E2 plays a very important role [6,7]. Previous studies have demonstrated that the E2 enzyme ubiquitin-conjugating enzyme E2D3 (UBE2D3) is involved in the regulation of cancer radiation resistance [8,9]. Another study has shown that ubiquitin-conjugating enzyme E2C (UBE2C) is highly expressed in many tumors and inhibition of UBE2C inhibits tumor progression [10]. Ubiquitin-conjugating enzyme E2T (UBE2T), a member of the E2 family, is located on human chromosome 1q32.1 and has a characteristic conserved domain with a size of about 16–18 kDa [11]. According to previous reports, UBE2T was used as an important member of the Fanconi signaling pathway to participate in DNA damage repair [12]. Recent studies have discovered that UBE2T is significantly increased in hepatocellular carcinoma, gallbladder cancer, and gastric cancer, and its high expression is closely associated with the tumor size, metastasis, and poor prognosis, suggesting that UBE2T may have the potential to promote the proliferation, invasion, and metastasis of malignant tumors [13–15]. For instance, Ueki et al. displayed that UBE2T promoted the progression of breast cancer by degrading BRCA1 [16]. Moreover, Wang et al. clarified that UBE2T down-regulation suppressed osteosarcoma cell proliferation and metastasis via inhibiting the PI3K/Akt signaling pathway [17]. More importantly, increasing evidence has shown that UBE2T is closely related to non-small cell lung cancer progression [18,19]. However, the correlation between UBE2T and LUAD, especially with regard to proliferation, invasion, migration, and apoptosis, has not yet been defined.

Fibulin-5 (FBLN5), a 66-kDa secreted glycoprotein, is identified by two independent groups in 1999 [20]. It has been reported that FBLN5 plays an important role in cell adhesion and motility, cell growth, cell metastasis, and tumorigenesis [21–23]. There is increasing evidence that FBLN5 has prognostic potential as a tumor suppressor in a variety of cancers, such as ovarian cancer, breast cancer, and hepatocellular carcinoma [24–26]. In lung cancer, overexpression of FBLN5 suppressed cell invasion and metastasis through the ERK pathway [27]. Another report demonstrated that FBLN5 impedes Wnt/β-catenin signaling by inhibiting ERK activation of GSK3β in lung cancer [28]. Furthermore, a previous report showed that ERK/GSK3β pathway regulates cell proliferation and metastasis and is frequently activated in tumor tissues including LUAD [29]. Besides, UBE2T was reported to promote the activation of GSK3β pathway in nasopharyngeal carcinoma [30]. However, whether FBLN5/ERK/GSK3β pathway was affected by UBE2T in LUAD is not clarified.

In this study, we hypothesized that UBE2T knockdown exerted an inhibitory effect on the progression of LUAD through regulating FBLN5 expression and ERK/GSK3β signaling pathway. The purpose of this study was to elucidate the functional role of UBE2T in the proliferation and metastasis of LUAD *in vitro* and *in vivo*, and explore the molecular mechanism underlying its role.

## Materials and methods

### Clinical samples

Sixty-five pairs of primary LUAD tissues and adjacent normal tissues were collected from patients admitted to the People’s Hospital of Shanxi Province, after receiving written informed consent. This study was approved by the Ethics Committee of People’s Hospital of Shanxi Province (approval no. SXSRM2018061325YY). This study was conducted following the ethical standards of our hospital and the Helsinki Declaration. The main clinical characteristics of the patients are summarized in Table 1.

**Table 1.** Correlations of UBE2T with clinicopathological features of LUAD

		UBE2T		
Item	*n*	High (*n* = 32)	Low (*n* = 33)	*p* Value
Age (years)				0.543
<60	24	13	11	
≥60	41	19	22	
Gender				0.536
Female	32	17	15	
Male	33	15	18	
Tumor size (cm)				0.165
<5	42	18	24	
≥5	23	14	9	
Local invasion				0.005*
T1-2	44	17	27	
T3-4	21	15	6	
Lymph node metastasis				0.035*
N0	35	13	22	
N1-3	30	19	11	
TNM stage				0.008*
I–II	41	15	26	
III–IV	24	17	7	

Statistical analyses were performed by χ^2^ test. *p < 0.05 was considered significant.

### Online database analysis

The analysis of UBE2T and FBLN5 levels in LUAD tissues from TCGA dataset was performed by using Gene Expression Profiling Interactive Analysis (GEPIA, http://gepia.cancer-pku.cn) [31]. The GEPIA and PrognoScan database (http://www.abren.net/PrognoScan) were applied to investigate the relationship between UBE2T and the prognosis of LUAD patients.

### Cell lines and cell culture

The lung adenocarcinoma cell lines (H1975 and H1650) and normal human bronchial epithelial cell line (HBE) used in this study were purchased from the Cell Bank of the Chinese Academy of Sciences (Shanghai, China). All the cells were cultured in DMEM with 10% FBS and maintained in an incubator at 37°C under 5% CO_2_ conditions [32].

### Generation of stable knockdown cell lines

The lentiviral vectors containing shRNA constructs for UBE2T, synthesized by Vigene Biosciences Inc. (Shanghai, China), were applied to knock down the endogenous UBE2T expression (sh-UBE2T-1, 5’-TTGTCTGGATGTTCTCAAATT −3’; sh-UBE2T-2, 5’-GCTGCTCATGTCAGAACCCAA-3’; sh-UBE2T-3, 5’-TGAC ATATCCTCAGAATTTAA-3’). FBLN5 shRNA was used to decrease FBLN5 expression (sh-FBLN5, 5’-CUGGUUUUACCCUCAAUGA-3’). The lentivirus vectors and scramble-negative control shRNA (sh-NC) were transfected into H1975 and H1650 cells, respectively, according to the manufacturer’s introductions. 96 h later, the puromycin was transfected into the infected cells to select UBE2T or FBLN5 stably silenced LUAD cells. The shRNAs cell lines with stable knockdown were measured by qRT-PCR [33].

### RNA extraction and quantitative real-time PCR (qRT-PCR)

Total RNA was extracted using RNAiso reagent (TaKaRa, Dalian, China) and reverse-transcribed to cDNA using PrimeScript RT Master Mix Kit (Takara) following the manufacturer’s instructions [34]. The reaction system was configured following the protocol of the SYBR Premix Ex TaqTM II kit (Thermo Fisher Scientific, Inc.), and the RNA transcript levels were performed using the Bio-rad CFX96 real-time PCR system (Biorad, USA). β-Actin was used as the internal control, and relative expression levels were calculated by the 2− ΔΔCt method. Primer sequence was shown as following: UBE2T-F-: 5’-TTGATTCTGCTGGAAGG ATTTG-3’; UBE2T-R: 5’-CAGTTGCGATGTTGAGGGAT-3’; FBLN5-F: 5’-CTGT GACCCAGGATATGAACTT-3’; FBLN5-R: 5’-TTGTAAATTGTAGCACGTCTGC- 3’; β-actin-F: 5’-TGGCACCC AGCACAATGAA-3’; β-actin-R-: 5’-CTAAGTCATA GTCCGCCTAGAAG CA-3’.

### Western blotting

Total protein was extracted from LUAD cells using RIPA buffer (Beyotime, Beijing, China) containing protease inhibitor and phosphatase inhibitor. The protein concentrations were detected by BCA assay (Beyotime, Beijing, China). An equal amount of protein was separated by 10% sodium dodecyl sulfate polyacrylamide gel electrophoresis (SDS-PAGE) and then transferred to polyvinylidene difluoride (PVDF) membranes (Millipore, CA, USA). After blocking with 5% skimmed milk for 2 h, the membranes were incubated with primary antibodies specific for UBE2T (1:1000, ab140611, Abcam), FBLN5 (1:500, ab66339, Abcam), Bcl-2 (1:2000, ab182858, Abcam), Bax (1:1000, ab32503, Abcam), cleaved-caspase-3 (1:500, ab32042, Abcam), pro-caspase-3 (1:1000, ab32499, Abcam), p-ERK (1:2000, Cell Signaling Technology, #4370), ERK (1:1000, Cell Signaling Technology, #4695), p-GSK3β (1:2000, ab75814, Abcam), GSK3β (1:2000, ab32391, Abcam), β-catenin (1:1000, Cell Signaling Technology, #8480), β-actin (1:1000, ab8227, Abcam) at 4°C overnight, followed by HRP-conjugated secondary antibody (1:2000, ab205718, ab6789, Abcam) for 1 h. The positive bands were detected by using an Enhanced Chemiluminescence Kit (Thermo Fisher Scientific) [32].

### Cell Counting Kit-8 (CCK-8) assay

For this, 5 × 10^3^ cells/well lentivirus infected LUAD cells were plated into 96-well plates. After incubation for 24, 48, 72, and 96 h, 10 μL of CCK-8 solution (5 mg/mL, Sigma) was added and incubation for another 2 h. The optical density values were then measured at a wavelength of 450 nm using a microplate reader (BioTek Instruments, USA) [34].

### Edu immunoflurescence assay

For this, 4 × 10^3^ cells/well LUAD cells were plated in a 96-well plate. After 24 h, the medium containing 50 mM Edu (100 mL) was added and incubated for 2 h at 37°C. Subsequently, the cells were fixed with 4% paraformaldehyde for 30 min and counterstained with Hoechst 33,342 for 10 min to stain the nucleus. The Edu-positive cells were counted under a fluorescence microscope (AF6000, Leica, Wetzlar, Germany) [35].

### Transwell assay

Stable expression LUAD cells (1 × 10^5^ cells/well) in serum-free media were placed into the upper chamber of an insert for migration assays (8-μm pore size, Corning, NY, USA) and invasion assays with Matrigel (Sigma-Aldrich, USA). The lower chambers were filled with complete medium supplemented with 20% FBS. After incubation for 48 h, the migrated or invaded cells were fixed with methanol for 10 min and stained with 0.1% crystal violet [32]. The cells were counted under a BX53 microscope in five randomly selected fields (Olympus, Japan) (magnification; 200×).

### TUNEL staining

One Step TUNEL Apoptosis Assay Kit (Beyotime) was applied to measure cell apoptosis according to the manufactures protocol [36]. Briefly, LUAD cells were incubated with PBS containing 0.3% Triton X-100 for 10 min and then incubated with 0.3% H_2_O_2_ in PBS for 20 min. Subsequently, the cells were incubated with TUNEL detection solution (50 μL) in the dark at 37°C for 1 h, followed by the streptavidin -HRP working solution for 30 min. Next, the cells were stained with Hoechst 33,342 for 10 min, and photographed by a fluorescence microscope (Fluoview FV1000, Tokyo, Japan) and counted by a Nikon ECLIPSE Ti fluorescence microscope under five random fields. Cell apoptosis (%) was calculated by the percentage of TUNEL-positive cells in the total number of cells (DAPI-positive cells).

### Chromatin immunoprecipitation (ChIP) assay

SimpleChIP® Plus Enzymatic Chromatin IP Kit (Magnetic Beads, CA, USA) was used to perform ChIP assay according to the manufacturer’s introduction [35]. In brief, LUAD cells were immobilized with formaldehyde, and the chromatin was fragmented by enzymatic hydrolysis and ultrasonic treatment. Subsequently, the chromatin was immunoprecipitated with specific anti-UBE2T, anti-FLBN5, and normal IgG antibodies. The enrichment of specific DNA fragments was analyzed by qRT-PCR.

The primers were as follows: Forward: 5’-ATCCCTCAACATCGCAACTGT-3’; Reverse: 5’-CAGCCTCTGGTAGATTATCAAGC-3’.

### Electrophoretic mobility shift assay (EMSA)

Biotin end-labeled probes were prepared by Sangon Biotechnology Co., LTD. (China). LightShift® Chemiluminescent EMSA Kit (Pierce, USA) was carried out to perform EMSA following the manufacturer’s instructions [37]. DNA binding reactions were performed with or without anti-UBE2T antibody. DNA–protein complexes were separated by electrophoresis and then transferred onto a positive-charged nylon membrane (Millipore, USA), followed by UV light crosslinking. The signal was visualized with chemiluminescent substrate followed by film exposure.

### Glutathione *S*-transferase (GST) pull-down assay

GST-UBE2T protein or GST control was transformed into *E. coli* BL21, and then 1 mmol/L IPTG was added to induce the protein expression [38]. Flag-FBLN5 protein was extracted from H1975 cell lysates. After GST-UBE2T and GST beads were cultured for 3 h, the eukaryotic expression protein Flag-FBLN5 was added to the mixture and the column was rotated vertically on the mixer for 3 h. Subsequently, the protein mixture was washed five times and denatured in 2× loading buffer at 95°C for 5 min. Protein bands were detected by western blotting.

### Tumor growth in vivo

A total of 20 female BALB/c nude mice (6–8 weeks old) were purchased from the Animal Center of the Chinese Academy of Science (Beijing, China). All animal experiments were approved by the Animal Care and Use Committee of the above hospital (approval no. SXSRM2019010264YY). H1975 cells stably expressing sh-UBE2T1 or negative control (sh-NC) were subcutaneously injected into the right flank of mice (2 × 10^7^ cells/mL, 0.2 mL, n = 5 in each group). The tumor volumes were recorded every 7 days (volume = length × width^2^)/2. Animals were euthanized via 2% pentobarbital sodium (120 mg/kg bodyweight) at 28 days, and then the tumors were peeled carefully and weighted [35].

### Immunohistochemical (IHC) analysis

The slides (4 μm-thick) of paraffin-embedded xenograft tissues were placed in xylene and ethanol for hydration treatment. After washing 3 times with PBS, the slides were completely immersed in 95°C antigen retrieval solution for 10 min. Then, 3% H_2_O_2_ were added and incubated for 10 min. After blocking with 5% serum for 30 min at 37°C, the slides were probed with specific rabbit anti-UBE2T antibody, mouse anti-FBLN5 antibody and rabbit anti-Ki67 at 4°C overnight, followed by the HRP goat anti-rabbit/mouse IgG for 1 h. Thereafter, DAB dropwise to the slides, and the color reaction was terminated with tap water. Finally, the slides were photographed by Olympus BX40 microscope (Tokyo, Japan) and quantified with Image ProPlus (IPP) software (Media Cybernetics, Rockville, MD, USA) [32].

### Statistical analysis

Statistical analysis was performed by using GraphPad Prism 8.0.2. Two-tailed unpaired Student’s *t* test and Turkey’s post hoc tests in one-way ANOVA were applied to analyze the differences between two groups or among the multiple groups. The χ^2^ test was used to evaluate the association between the expression of UBE2T1 and clinicopathological characteristics of LUAD patients. All data are shown as the mean ± SD. *P* < 0.05 was considered as a statistically significant.

## Results

This study was aimed to elucidate the functional role of UBE2T in the proliferation and metastasis of LUAD *in vitro* and *in vivo* and to explore the molecular mechanism underlying its role. Results showed that UBE2T was significantly elevated in LUAD tissues and high UBE2T expression was associated with poor overall survival. Results from the loss-of-function experiments *in vitro* showed that UBE2T modulated LUAD cell proliferation, migration, invasion, and apoptosis. The mechanism analysis demonstrated that silence of UBE2T increased FBLN5 expression and inhibited the activation of ERK/GSK3β pathway. In *in vivo* experiments, it was found that UBE2T knockdown inhibits the tumor growth in accumulating evidence has shown that that FBLN5, as a tumor suppressor, has LUAD. These results suggested that UBE2T might be a potential biomarker of LUAD, and targeting the UBE2T/FBLN5 axis might be a novel treatment strategy for LUAD.

### High expression of UBE2T was closely related to the poor prognosis of LUAD patients

To determine the expression status of UBE2T in LUAD, the online tool GEPIA was applied to analyze TCGA LUAD dataset. Results revealed that the UBE2T mRNA expression was elevated markedly in LUAD tissues versus to that in normal tissues (Figure 1(a)). In addition, UBE2T expression was evaluated in 65 pairs of LUAD tissues. In line with TCGA dataset results, UBE2T was significantly upregulated in LUAD tissues in comparison with normal tissues (Figure 1(b)). Similarly, the protein level of UBE2T was increased in LUAD tissues (Figure 1(c)). Next, the relationship between UBE2T and the survival rates of LUAD patients was evaluated. According to the median level of UBE2T, patients were divided into low-expression group and high-expression group. Results displayed that high UBE2T expression was closely associated with the poor overall survival and poor disease-free survival in LUAD patients (Figure 1(d,e)). Another online database, PrognoScan database, was then used to examine the prognostic potential of UBE2T in LUAD. As shown in Figure 1(f,g), there was a poor prognosis in LUAD patients with high UBE2T expression than in those with low UBE2T expression. Therefore, these findings suggested that UBE2T might be a potential prognostic biomarker for LUAD patients.

**Figure 1.** High expression of UBE2T was correlated with poor prognosis of LUAD patients. (a) GEPIA analysis of UBE2T expression in LUAD tissues from TCGA dataset. (b) qRT-PCR analysis of UBE2T expression in 65 pairs of LUAD tumor tissues and adjacent non-tumor tissues. (c) UBE2T protein level analyzed by western blotting in four pairs of LUAD tumor tissues and adjacent non-tumor tissues. (d) GEPIA analysis of the correlation between UBE2T expression and overall survival from TCGA LUAD dataset. (e) GEPIA analysis of the relationship between UBE2T expression and disease-free survival from TCGA LUAD dataset. (f) The relationship between UBE2T expression and overall survival from the LUAD cohort (GSE31210, *n* = 204). (g) The relationship between UBE2T expression and disease-free survival from the LUAD cohort (GSE31210, *n* = 204). *p < 0.05.

### UBE2T knockdown suppressed LUAD progression

To investigate the functional roles of UBE2T in LUAD, UBE2T expression was first measured in LUAD cells. Results from qRT-PCR showed that UBE2T was higher in LUAD cells than that in normal human HBE cells (Figure 2(a)). H1975 and H1650 cells were infected with sh-UBE2T and sh-NC. qRT-PCR results showed that UBE2T was down-regulated in sh-UBE2T LUAD cells versus to that in control group (Figure 2(b)), sh-UBE2T-1 was selected for further experiments for its stronger inhibitory effects. CCK-8 assays displayed that the proliferation rate of H1975 and H1650 cells treated with sh-UBE2T-1 was slower than that with sh-NC (Figure 2(c)). Edu assays showed that UBE2T knockdown decreased the percentage of Edu-positive cells in comparison with control group (Figure 2(d)). Transwell migration assay discovered that H1975 and H1650 cells with sh-UBE2T-1 had less migrated cells than that of cells with sh-NC (Figure 2(e)). Moreover, results from transwell invasion assay revealed that H1975 and H1650 cells with sh-UBE2T-1 had less invasive cells than that of cells with sh-NC (Figure 2(f)). Besides which, western blotting assay discovered that Bcl-2 level was down-regulated, while Bax and cleaved-caspase-3 levels were upregulated in sh-UBE2T-1 LUAD cells, relative to sh-NC group (Figure 2(g)). Meanwhile, TUNEL staining revealed that the apoptosis cells was obviously increased in sh-UBE2T-1 group (Figure 2(h)). These data indicated that UBE2T knockdown inhibited LUAD cell proliferation, migration, invasion, and promoted cell apoptosis.

**Figure 2.** UBE2T knockdown inhibited LUAD progression. (a) qRT-PCR analysis of UBE2T mRNA expression in LUAD cells and normal human HBE cells. (b) qRT-PCR analysis of UBE2T expression in H1975 and H1650 cells transfected with sh-UBE2T. (c) CCK-8 assays analysis of cell viability of H1975 and H1650 cells with sh-UBE2T-1. (d) Cell proliferation of H1975 and H1650 cells with sh-UBE2T-1 was measured by Edu assay (Scale bar = 50 mm). (e) Measurement of the migration of H1975 and H1650 cells with sh-UBE2T-1 by transwell assay (×200 magnification). (f) Measurement of the invasion of H1975 and H1650 cells with sh-UBE2T-1 by transwell assay (×200 magnification). (g) Detection of Bax, Bcl-2, cleaved-caspase-3 and pro-caspase-3 levels in H1975 and H1650 cells with sh-UBE2T-1 by western blotting. (h) Detection of the apoptosis of H1975 and H1650 cells with sh-UBE2T-1 by TUNEL staining assay (scale bar = 50 mm). *p < 0.05, **p < 0.01, ***p < 0.001.

### UBE2T knockdown contributes to the increase of FBLN5 and inactivation of ERK/GSK3β pathway

To investigate the underlying mechanism of UBE2T in LUAD, cBioPortal database (https://www.cbioportal.org) was applied to search for UBE2T-related genes. Among those genes, FBLN5 was a negatively correlated gene of UBE2T in LUAD *r* = −0.54, *p* = 0.0124, Figure 3(a). Besides, GEPIA with the Spearman correlation test showed a negative correlation of UBE2T with FBLN5 mRNA expression *r* = −0.45, *p* < 0.001, Figure 3(b). In addition, the relationship between UBE2T and FBLN5 expression was evaluated in LUAD tissues as well. In line with the online database results, UBE2T was negatively correlated with FBLN5 in LUAD tissues (Figure 3(c)). Furthermore, the effect of UBE2T on FBLN5 activity was investigated in LUAD. qRT-PCR results displayed that UBE2T knockdown increased FBLN5 expression in LUAD cells (Figure 3(d)). Similarly, results from western blotting revealed that UBE2T down-regulation increased the level of FBLN5 (Figure 3(e)). Importantly, ChIP-qPCR assays displayed that UBE2T enhanced the enrichment of FBLN5 in LUAD cells (Figure 3(f)). A subsequent EMSA discovered that when the native probe was incubated with purified UBE2T protein, a DNA-protein complex was formed, and the mutated probe reduced the binding capacity. An antibody supershift assay further verified that UBE2T directly bound to native probe (Figure 3(g)). In addition, results from GST pull-down assay demonstrated that there was a direct interaction between GST-UBE2T and Flag-FBLN5 (Figure 3(h)). These results indicated that FBLN5 might be a potential target gene of UBE2T in LUAD. Next, the expression status of FBLN5 was determined in LUAD, TCGA database results displayed that FBLN5 was significantly decreased in LUAD tissues, relative to that in normal tissues (Figure 3(i)). Furthermore, in our own cohort, FBLN5 was obviously reduced in LUAD tissues, when compared to normal tissues (Figure 3(j)). Western blotting results discovered that compared with sh-NC LUAD cells, the levels of p-ERK, p-GSK3β, and β-catenin were down-regulated in LUAD cells with sh-UBE2T-1 (Figure 3(k)). These findings suggested that UBE2T knockdown suppressed the activation of ERK/GSK3β pathway in LUAD.

**Figure 3.** UBE2T knockdown contributes to the increase of FBLN5 and inactivation of ERK/GSK3β pathway. (a) The relationship between UBE2T and FBLN5 expression from cBioPortal database was analyzed by Spearman correlation analysis. (b) The relationship between UBE2T and FBLN5 expression from TCGA dataset was analyzed by GEPIA. (c) The relationship between UBE2T and FBLN5 expression was analyzed by Spearman correlation analysis using 65 LUAD tissues. (d) qRT-PCR analysis of FBLN5 expression in H1975 and H1650 cells with sh-UBE2T-1. (e) Western blotting analysis of FBLN5 level in H1975 and H1650 cells with sh-UBE2T-1. (f) ChIP–qPCR showed the association of FBLN5 with UBE2T in LUAD cells. (g) An EMSA and a supershift assay showed that UBE2T bound to the FBLN5 promoter. (h) GST pull-down demonstrated a direct interaction between GST-UBE2T and Flag-FBLN5. (i) GEPIA analysis of FBLN5 expression in LUAD tissues from TCGA dataset. (j) qRT-PCR analysis of FBLN5 expression in 65 pairs of LUAD tumor tissues. (k) Measurement of p-ERK, ERK, p-GSK3β, GSK3β, β-catenin levels in H1975 and H1650 cells with sh-UBE2T-1 by western blotting. *p < 0.05, **p < 0.01, ***p < 0.001.

### FBLN5 knockdown abrogated the inhibitory effect of sh-UBE2T on LUAD progression

Given that UBE2T modulated LUAD cell proliferation and metastasis and regulates FBLN5 expression in LUAD cells, the effect of FBLN5 on UBE2T-regulated cell proliferation and metastasis was further explored. H1975 and H1650 cells were transiently transfected with sh-NC, sh-UBE2T-1, or sh-UBE2T-1+ sh-FBLN5. Results from CCK-8 showed that H1975 and H1650 cells with sh-UBE2T-1 exhibited a decrease in the cell viability and FBLN5 depletion partially reversed sh-UBE2T-inhibited cell viability (Figure 4(a)). Meanwhile, Edu assay results discovered that the positive cells generated in sh-UBE2T-1+ sh-FBLN5 groups were notably enhanced versus to that in sh-UBE2T-1 group (Figure 4(b)). Moreover, results of Figure 4(c) show that the decrease in the migration resulting from UBE2T knockdown was partially rescued by silence of FBLN5. Similarly, as shown in Figure 4(d), there was a significant decrease in invasion abilities in UBE2T knockdown cells, and the decrease was restored by combining with FBLN5 inhibition (Figure 4(d)). In addition, western blotting revealed that sh-UBE2T-1 remarkably reduced Bcl-2 level and accelerated Bax and cleaved-caspase-3 levels in LUAD cells, which were partially overturned by combining with FBLN5 depletion (Figure 4(e)). TUNEL assay manifested that the promotion effect of sh-UBE2T-1 on LUAD cell apoptosis was also partly attenuated by the combined with sh-FBLN5 (Figure 4(f)). Collectively, these results confirm that knockdown of UBE2T suppressed the proliferation and metastasis potential possibly by activating FBLN5 expression in LUAD cells.

**Figure 4.** FBLN5 knockdown abrogates the inhibitory effect of sh-UBE2T on LUAD progression. (a) sh-FBLN5 partially reversed sh-UBE2T-1-inhibited viability in H1975 and H1650 cells, as measured by CCK8 assay. (b) sh-FBLN5 partially reversed sh-UBE2T-1-inhibited proliferation in H1975 and H1650 cells, as measured by Edu assay. (c) FBLN5 inhibition abrogated sh-UBE2T effect on migration and (d) invasion, as measured by transwell assay (×200 magnification). (e) FBLN5 depletion overturned the effect of sh-UBE2T on Bax, Bcl-2, and cleaved-caspase-3 levels, as measured by western blotting. (f) sh-FBLN5 partially attenuated sh-UBE2T-1-enhanced apoptosis in LUAD cells, as measured by TUNEL assay (Scale bars = 50 μm). *p < 0.05, **p < 0.01; #*p* < 0.05.

### UBE2T knockdown inhibited tumor growth in vivo

To determine the effect of UBE2T on LUAD *in vivo*, H1975 cells with sh-UBE2T-1 were injected into nude mice to establish xenograft tumor models. Twenty-eight days after inoculation, the mice were euthanized and dissected (Figure 5(a)). The tumor volume and tumor weight were remarkably down-regulated in the sh-UBE2T-1 group compared to sh-NC group (Figure 5(b,c)). IHC results showed that the tumor cell proliferation marker Ki67 was decreased in the sh-UBE2T-1 group, relative to the control group (Figure 5(d)). Moreover, UBE2T was obviously decreased, while FBLN5 was increased in the tumor tissues of sh-UBE2T-1 group compared with sh-NC group (Figure 5(e,f)). These results indicated that UBE2T knockdown inhibited LUAD tumor growth *in vivo*.

**Figure 5.** UBE2T knockdown suppressed tumor growth *in vivo*. (a) Photograph of tumors at 28 days after transplantation. (b) Measurement of tumor volume every 7 days, and plots of growth curves. (c) Measurement of tumor weight at 28 days after transplantation. (d) The expression of Ki67, (e) UBE2T, and (f) FBLN5 in tumor tissues with sh-UBE2T-1, as measured by IHC assay (scale bar = 25 μm). *N* = 4 for each group. **p < 0.01.

## Discussion

The dysregulation of UBE2T is closely related to the occurrence and development of various tumors [39,40]. Although a previous study has shown that UBE2T was elevated markedly in non-small cell lung cancer tissues and ranked first according to the hazard ratio in the survival analysis [18], the functional role and molecular mechanism of UBE2T in LUAD proliferation and metastasis remain unknown. Herein, we discovered that UBE2T was upregulated in LUAD tissues in TCGA dataset, as well as in LUAD tissues and cells. The results were similar to the previous study that UBE2T was over-expressed in lung cancer, which was confirmed by western blotting, qRT-PCR, and immunohistochemistry [41]. Notably, analyzing TCGA survival data and PrognoScan database demonstrated that high UBE2T expression strongly indicated poor prognosis of LUAD patients. Collectively, these findings indicated that UBE2T might be a promising biomarker for the prognosis and diagnosis of LUAD patients. Moreover, the loss-of-function assay results revealed that UBE2T knockdown suppressed LUAD cell proliferation, migration, and invasion *in vitro* and tumor growth *in vivo*. Taken together, these findings revealed that UBE2T exhibited the critical oncogenic roles in LUAD and UBE2T was indicated as a potential therapeutic target for LUAD.

ChIP-qPCR assay, EMSA assay, GST pull-down assay, and TCGA data analysis were applied to explore the mechanisms of UBE2T in LUAD. Through cBioPortal database and TCGA data analysis, the potential targets of UBE2T were screened. Among those genes, FBLN5 may be a possible factor involved in the development of LUAD. FBLN5, an extracellular matrix protein, takes part in regulating the proliferation, invasion and angiogenesis of malignant tumor cells [2–3]. It has been reported that FBLN5 was significantly down-regulated in ovarian cancer [24], breast cancer [42], and lung cancer [28], and FBLN5 over-expression inhibited cells proliferation and metastasis. In line with previous results, the analysis of online databases and our findings discovered that FBLN5 was down-regulated in LUAD tissues, and statistical analysis showed a negative relationship between UBE2T and FBLN5 expression. Our findings also displayed that UBE2T knockdown activated FBLN5 expression by qRT-PCR, western blotting. Moreover, UBE2T bound to FBLN5, which was confirmed by ChIP-qPCR, EMSA and GST pull-down assays. The FBLN5 up-regulation might be crucial for UBE2T-mediated cell proliferation, migration and invasion. Thus, the effects of FBLN5 on UBE2T-regulated cell proliferation and metastasis was investigated. The rescue experiments revealed that the inhibitory effect of sh-UBE2T on the proliferation, migration, and invasion were reversed by sh-FBLN5.

Given previous studies shown that FBLN5 was involved in lung cancer development via the ERK pathway. A recent study showed that p-ERK promotes β-catenin activity by suppressing its regulatory molecule GSK3β [43]. Our study demonstrated that silence of UBE2T decreased the levels of p-ERK, p-GSK3β, and β-catenin, indicating that UBE2T knockdown impeded the activation of ERK/GSK3β signaling pathway.

There are limitations in this present study. First, only H1975 cells used in *in vivo* experiments, due to the limitation of time and technology. Second, the mechanisms of LUAD are complex and the targets of UBE2T are diverse; several crosstalk signaling pathways participate in the network regulated by UBE2T in LUAD, it is necessary to further study how UBE2T regulates FBLN5 and ERK/GSK3β signaling pathway. Third, there are few clinical research in this paper, which should be performed in further studies.

## Conclusions

This present study showed that UBE2T deficiency suppressed LUAD progression through increasing FBLN5, and suppressing the activation of ERK/GSK3β pathway. These results elucidate the underlying mechanism by which UBE2T regulates LUAD progression and provides a new direction for the development of effective treatment strategies for LUAD.

## Data Availability

The datasets used and/or analyzed during the present study are available from the corresponding author on reasonable request.
